The article "Application Model of Public Health Visual Art Creation Concept Based on Artificial Intelligence Technology in Venice Biennale" was retracted in 2023. Reasons: unreliable results or conclusions; concerns about the data; concerns about the results or conclusions; concerns about the peer review.

# Application Model of Public Health Visual Art Creation Concept Based on Artificial Intelligence Technology in Venice Biennale

**DOI:** 10.1155/2022/6546357

**Published:** 2022-09-05

**Authors:** Xiaohe Xie

**Affiliations:** School of Art, Southeast University, Nanjing 21000, China

## Abstract

There are some problems in the creation process of public health visual art works, such as low accuracy and poor content quality. In order to further improve the accuracy and quality of artistic creation, based on artificial intelligence technology, a neural network model and an error backpropagation algorithm are used to analyze artistic creation, so as to obtain the corresponding optimization model. This model can analyze the application of public health visual art creation concepts in the Venice Biennale, so as to obtain the corresponding model calculation results under different indicators. Finally, data comparison is used to verify the accuracy of the model. Relevant studies show that activation values have different trends in connection weights under the action of different factors. The fluctuation of the curve is obvious in the initial state, but when the factor is high, the corresponding connection weight tends to be stable gradually. The range of learning rate in the initial state is relatively small, and the connection weights show a V-shaped change at higher factors. It can be seen from the curve corresponding to the *ω* learning method that the increase in learning speed will lead to further compression of calculation time, and the curve shows a trend of fluctuation. The corresponding learning error decreases gradually with the increase in factors, which indicates that higher factors will promote the accuracy of connection weights. Artificial intelligence-based visual models of art can calculate public health. It can be seen from the calculation results that the curve corresponding to artistic connotation has the largest range of variation and the highest influence on the model. The theme, form, and style of art all show a linear trend of improvement with the increase in time, while the content of art shows a downward trend. This research can provide support for the application of artificial intelligence theory in the field of public health.

## 1. Introduction

Artificial intelligence plays an important role in many fields, such as clinical medical diagnosis [1], college English education [2], enterprise management [3], and technology mining [4]. In view of the problems existing in the industrial design system such as complex operation, a deep learning method was adopted to analyze the industrial design data based on artificial intelligence technology, so as to obtain the data change rule under different indicators. It was introduced into the original model for optimization, so as to obtain the corresponding optimization model [5]. The model can analyze industrial design under different design methods, and conduct targeted research on industrial design through data extraction, algorithm calculation, and model verification. As an important form of classroom teaching, the wisdom classroom was playing an increasingly important role. In order to solve the problems existing in the classroom, based on the artificial intelligence technology, the neural network and the fuzzy set calculation methods were used to extract the data in the classroom. The optimal solution of classroom teaching was found through calculation and analysis [6], which can provide theoretical support for the promotion of smart classroom. Finally, experimental data were used to verify the accuracy of the model.

In view of the problems existing in the creation process of public health visual art works, based on artificial intelligence technology, the neural network computing method was used to extract the data, so as to obtain the corresponding optimization model. Then, the application model of art creation under the theory of artificial intelligence was established, and the model was applied to the Venice Biennale; the corresponding calculation results were obtained through calculation. Finally, the accuracy of the model was verified by the method of experimental comparison. The research shows that the model can provide ideas and concepts for the creation of art works.

## 2. Artificial Intelligence Technology

Artificial intelligence technology is also known as machine intelligence [7, 8]. Usually, artificial intelligence refers to human intelligence technology achieved by means of ordinary computer programs. Artificial intelligence technologies include machine learning, machine vision, robotics, natural language processing, and automation [9, 10].

Artificial intelligence is playing an important role in creating public health art. In order to further study its creation process in the field of public health, the training process under the effect of the neural network was obtained by summarizing and analyzing relevant visual art works, as shown in Figure 1. The neural network training process based on artificial intelligence is as follows: firstly, the data are initialized and analyzed, and then, the data obtained from initialization analysis are imported into the output parameters. The structure and type of grid are determined by the output parameter module, and then introduced into the input vector module for the corresponding target output. According to the obtained target output results, it is imported into the hidden layer for corresponding result output, so as to obtain the comparison between the target value and the actual error. Through the assumption judgment, it can be seen that if it meets the requirements of maximum training times, the corresponding calculation process shall be derived; and that if it does not meet the requirements of maximum training, the data shall be further analyzed for error requirements. The error requirement module further determines the difference between all errors and partial errors, calculates the error between the corresponding units, imports it into the correction weight, and then outputs the corresponding data.

### 2.1. Basic Model of Neural Network

A large number of simple neurons form a relatively complex neural network, with several inputs and unique outputs for each neuron [11, 12]. Each neuron in the neural network is connected by variable weights. The artificial neural network composed of a large number of neurons can be regarded as a directed graph, and each neuron connection corresponds to a real number, namely, the connection weight coefficient, or weight. The set of weights can act as a long-term memory and change dynamically. During the training of the neural network, the weights of connections between neurons are constantly changed in the training process. The relationship between input vector and output vector is as follows:

(1) $$\begin{array}{c} y=f\left(\sum_{i=1}^{m}w_{i}x_{i}-\theta \right), \end{array}$$

where *θ* is the threshold value and *f*(*x*) is the excitation function. Commonly used excitation functions include step function, piecewise function, and Sig function. In the multilayer neural network, there is a functional relationship between the output of the upper node and the input of the lower node, which is called the activation function. The advantages of the excitation function are mainly reflected in the following: (1) it can adjust the proportion of input to output or effectiveness; (2) it can convert input and output; and (3) it can be realized to constrain an infinite set to a finite specified range.

The excitation function plays an important role in the calculation of the neural network basic model. In order to further analyze the relationship between the output vector and the input vector, it can be seen from the analysis that the threshold value and the excitation function will have a great influence on the results of the output value. In order to further analyze the influence rule between the threshold value and the excitation function, the change curve of the excitation function was obtained through calculation, as shown in Figure 2. It can be seen from the figure that the threshold value and the excitation function have different changing trends under the action of different input values: firstly, it can be seen from the change of the threshold value that the curve increases gently at first, then further increases with the increase in input value, and the curve rapidly jumps to the local maximum value. In the linear increase stage, the slope of the curve is relatively low, and when the output value exceeds the local maximum value, the curve drops rapidly to the local minimum value. With the further increase in the input value, the curve rapidly increases to the maximum value. The curve as a whole shows a gradual increasing trend of change. For the corresponding excitation function, the increase in input value shows a linear change trend of gradually decreasing to the local lowest point first and then increasing rapidly. The change in the first stage of the curve shows a V-shaped change as a whole. Then, as the input value increases, the curve overflows smoothly before gradually falling to its lowest point. It can be seen from the analysis that the threshold value and the excitation function have different changing trends, and the corresponding relationship between the input value and the output value can be well reflected by the change of the two data.

Common mathematical models of neural networks are shown as follows: (1) interconnection artificial neural networks: in the process of network training, the whole neural network is optimized by constantly updating the weights of connections between neurons. The interconnected artificial neural network is constantly optimized in the training process to get the corresponding calculation results. After a period of time, the neural network can reach a relatively stable state. The biggest advantage of this type of neural network is that there are connections between each neuron, which can make the neural network training reach a better state. The biggest disadvantage is the slow speed of network training; (2) feedforward artificial neural network, in which neurons are arranged hierarchically, is a one-way transmission network model with input and output signals. The model is composed of three layers, the first layer is the input layer, the middle layer is the hidden layer, and the last layer is the output layer. Each neuron can take input from one layer and send output to the next, and so on. Different from interconnected neural networks, feedforward neural networks have no reverse transfer from lower layer to upper layer; and (3) feedback forward network: the input layer neurons in the network continuously receive feedback input from the output layer neurons or some of the output layer neurons in the learning process, and feedback the output of the network to the input of the network.

### 2.2. Artificial Neural Network

The core research problem of the artificial neural network is its learning method. When the topology structure of the neural network is determined, the intelligent characteristics of the neural network can only be made by selecting appropriate learning methods and combining with the topology structure [13, 14]. The learning method of the artificial neural network is to adjust the connection weights of each neuron in the network. Every functional area of the human brain has clever and perfect learning rules; different functional areas have different learning rules. These rules are learned and refined over time through the evolution of the human brain.

According to the function and structure of the neural network, the corresponding learning methods have different forms [15, 16]. These learning methods have their own advantages for solving all kinds of problems [17, 18]. The following is a brief introduction to some common learning rules in artificial neural networks:

(1) Hebb's learning rule: when two adjacent neurons are activated at the same time, this learning method can increase the connection weight between them. Hebb's learning method can be expressed as follows:
  (2) $$\begin{array}{c} \Delta w_{ij}=a\times vi\times vj, \end{array}$$
  where *vi* and *vj* are the activation values of the output function, respectively; *w*_*ij*_ is the connection weight of the neuron; and *a* is the network learning rate.
Hebb's learning rule is one of the most important learning rules in the artificial neural network. It can be seen from the above calculation formula that the activation function and learning rate corresponding to input value and output value will have a great influence on the model connection weight. In order to further analyze the change rule of activation value and learning rate under the action of different factors, the change curve of corresponding Hebb's learning rule was obtained through calculation, as shown in Figure 3. It can be seen from the curve of Hebb's learning rules that the activation value shows a trend of gradual increase with the gradual increase in factors, with a relatively small fluctuation range and an approximate linear change trend as a whole. However, due to the jump of other factors in the data, the corresponding connection weight fluctuates in the lower range of factors. When it is under the action of higher factors, the curve increases rapidly and then transitions smoothly. This shows that the effect of the activation function on the total value of the connection has a positive linear distribution characteristic. It can be seen from the curve of learning rate that with the gradual increase in factors, the curve first slowly increases and then rapidly decreases, and then rapidly increases to the maximum value and then gradually decreases. This indicates that the learning rate has a relatively small impact on the connection weight and the overall fluctuation range of the curve is relatively small.
The weight connection rules of the artificial neural network show different changes according to different calculation contents. The adjustment of connection weights between various neurons in the current artificial neural network can be roughly divided into two rules: one is to get specific weights directly through calculation, and the other is to optimize and improve the neural network after continuous learning.
(2) *ω* learning method: this is a learning method with known sample results. *X* is taken as the input vector of the neural network, and the network output vector *Y* is obtained under the joint action of the connection weights between each neuron [19]. The essence of the *ω* learning method is to take the derivative of the quadratic error function, and its concrete implementation is a learning method of gradient derivation. The choice of function is based on the specific application. Learning rules are widely used, among which the most typical application is the algorithm of the feedforward neural network. The calculation formula of the weight adjustment range of this learning method is shown as follows:
  (3) $$\begin{array}{c} \Delta w_{ij}=a\times vi\times \omega j,\\ \omega j=F\times \left(yj-\bar{y}j\right), \end{array}$$
  where $\left(yj-\bar{y}j\right)$ is the learning error.
*ω* learning method is an important part of the artificial neural network calculation method and is mainly influenced by learning rate and learning error. The learning rate will affect the learning speed, and the learning error will affect the accuracy of the artificial neural network. In order to analyze the influence rules of these two factors, the change curve of learning methods is drawn through analysis, as shown in Figure 4. It can be seen from the curve that the learning speed increases linearly with the increase in factors, then decreases linearly to the lowest point, and then increases linearly. This indicates that the learning rate has a positive linear effect on the connection weights. At the same time, it can be seen from the learning error that with the gradual increase in factors, it shows a rapid decline at first and then gradually tends to a gentle trend. This indicates that the smaller the factor is, the larger the error of the artificial neural network model is. When the factor is higher and higher, the error of the curve connection weight is relatively small, but with the further increase in the factor, the error remains stable.
Connection weights can be divided into positive and negative cases. When it is positive, it means that the neuron is excited. When it is negative, it indicates that the neuron is inhibited. The training of the neural network is mainly reflected in the change of connection weight. The connection weights also describe the characteristics of neural networks.
(3) Similarity learning method: *w*_*ij*_ is the connection weight between network neuron *i* and network neuron *j*, *vi* is the output value of network neuron, and then, the connection weight between network neuron *i* and network neuron *j* is adjusted as follows:

(4) $$\begin{array}{c} \Delta w_{ij}=a\left(vi-w_{ij}\right). \end{array}$$

It can be seen from the formula that the accuracy of the learning rules is relatively high, and the corresponding learning methods are also widely used.

Similarity learning is an important part of the artificial neural network, which can further reflect the connection weights between neuron *i* and neuron *j*. The contour map corresponding to the similarity learning method can be obtained through analysis, as shown in Figure 5. It can be seen from the curve changes in the figure that the connection weights have different changing trends under the action of different factors. The learning rate increases gradually with the increase in factors, and the corresponding weight changes greatly under higher factors. It can be seen from the learning error that with the increase in factors, the corresponding connection weights show a trend of gradual increase, and the overall fluctuation range is relatively large. Based on the above analysis, it can be seen that two different factors have the same influence on the similarity learning method. Therefore, the influence of two factors should be comprehensively considered to obtain an accurate similarity learning method.

### 2.3. Theoretical Analysis of an Error backpropagation Algorithm

The error backpropagation algorithm (BP algorithm) is a kind of a guided learning algorithm, which is used to calculate network weights and thresholds [20, 21]. The main idea of weight learning of the BP neural network is to gradually determine the connection weight through two different directions: forward and reverse. It can be roughly described as follows: firstly, in the forward propagation process, there is an initial connection weight in the initial state of the neural network. Then, the model gradually propagates and processes through each hidden layer, calculates the actual output value of each neuron, and finally gets an output value. The algorithm contains a hidden layer feedforward network, which plays an important role in improving the classification ability of the neural network. The neural network system proposed by the algorithm solves the problem of learning the connection weights between hidden neurons in the neural network structure with multiple hidden layers [22, 23]. The neural network is the most widely used the neural network model. It is a typical forward feedback neural network. The network structure has an input layer and multiple hidden layers, each of which has a different number of nodes. For the input information of the input layer, it first passes through the input layer to the hidden layer, which may go through multiple hidden layers, and finally gives an output vector. In the process of information transmission, the final change of information is determined by the connection weights between the activation function and each neuron.

The BP algorithm is a kind of learning method based on a gradient layer-by-layer descent method, especially suitable for the network structure with multiple hidden layers [24, 25]. A large number of theories have proved that the neural network can approach any nonlinear function within the required error range through continuous training of the network. Now suppose that each neuron in a particular network has inputs from each neuron in the upper layer and outputs to each neuron node in the lower layer [26, 27]. The characteristic of each neuron is Sig type, which is continuously differentiable unlike the linear threshold function of perceptron. The corresponding calculation formula is as follows:

(5) $$\begin{array}{c} N=\sum_{j}wij\times Pik,\\ P_{1}ik=f\left(N\right), \end{array}$$

where *Pik* is the corresponding output result when the *k*-th sample is input and *N* is the actual output value of the model. The error function adopted is as follows:

(6) $$\begin{array}{c} Ek=\frac{1}{2}{\sum_{l}\left(yk-\bar{y}k\right)}^{2}, \end{array}$$

where *yk* is the ideal value of the neural network and $\bar{y}k$ is the actual output result.

Through the neural network basic model and the artificial neural network, the corresponding BP algorithm theory can be obtained. Through the above analysis, the corresponding calculation function of the output neural network can be obtained. Different models will have different influences on the calculation function. Therefore, in order to further study the influence of different parameters in the function on the dependent variable of the model, the change curves of different models under the action of independent variables are drawn, as shown in Figure 6. As can be seen from the figure, model value, sample value, ideal value, actual value, and other factors will have a great impact on the function. Through analysis, it can be seen that with the increase in the independent variable, the model value first presents a trend of gradual increase, then gradually decreases, then continues to increase to the maximum value, and finally gradually decreases. This indicates that the increase in independent variables will have a certain impact on the calculation results of the model, but the fluctuation range is relatively small. As can be seen from the sample value, it shows a linear increase trend with the increase in independent variable, while when the dependent variable reaches the local maximum value, the curve gradually tends to be gentle. When the value of the independent variable increases to the maximum, the corresponding curve shows a trend of gradual decline. From the ideal value, it can be seen that as the independent variable increases, the curve increases rapidly, and the slope of the corresponding curve is higher than that of the model value and the sample value, and then, the curve remains stable. When the independent variable increases gradually, the corresponding dependent variable also remains stable. As can be seen from the change curve corresponding to the actual value, the slope of the linear stage is the largest, and the increase in the independent variable will cause the actual value of the model to fluctuate to a certain extent first, and then show a phased decline. Through the above analysis, it can be seen that four different types of function variables have different influences on the dependent variables of the model. Therefore, the relationship between function model value, sample value, ideal value, and actual value should be considered comprehensively to obtain the corresponding output function.

The total error of the model function is as follows:

(7) $$\begin{array}{c} E=\frac{1}{2N}\sum_{k=1}^{N}Ek. \end{array}$$

The corresponding calculation formula of model weight modification variables is as follows:

(8) $$\begin{array}{c} W=wij-u\frac{\partial E}{\partial wij}. \end{array}$$

Through error and corresponding correction analysis of the above model functions, the corresponding model weight correction variable graph is obtained, as shown in Figure 7. It can be seen from Figure 7 that the revised data gradually increase over time, showing a trend of linear decline and a relatively large decline. As time goes on, the modified data fluctuate in a certain range, which indicates that there is a certain error in the corresponding calculation method at this stage, leading to varying degrees of fluctuation in the modified data. With the further increase in time, the curve shows an approximate V-shaped change; that is, the maximum value increases rapidly at first and then decreases rapidly. On the whole, the data have the characteristics of linear and nonlinear overall change. It can be seen from the corresponding correction curve that it can not only better describe the linear stage of the curve, but also better reflect the range of the fluctuation stage and the change of specific data. Therefore, it can be seen from the above model weight modification curve that the modification curve can better meet the changes of modified data.

In order to compare the prediction performance of each model, two model evaluation indexes were selected: mean square error and direction change statistics [28, 29]. The expression of mean square error is as follows:

(9) $$\begin{array}{c} \text{NMSE}=\frac{\sum_{t=1}^{N}{\left(y-\hat{y}\right)}^{2}}{\sum_{t=1}^{N}{\left(y-\bar{y}\right)}^{2}}=\frac{1}{N\sigma^{2}}\sum_{t=1}^{N}{\left(y-\hat{y}\right)}^{2}, \end{array}$$

where *y* is the actual value, $\hat{y}$ is the predicted value, and *σ*^2^ is the estimated error.

The expression of the direction change statistic is as follows:

(10) $$\begin{array}{c} D=\frac{1}{N}\sum_{t=1}^{N}at,\\ a=\left\{\begin{array}{c} 1,\left(y-\hat{y}\right)\left(y-\bar{y}\right)\geq 0,\\ 0,\text{other}. \end{array}\right. \end{array}$$

The neural network and model algorithm theory based on artificial intelligence technology can get different results [30, 31]. In order to further study the influence of different factors on the neural network, and then the effect of the results of artificial intelligence technology, two different model indexes are obtained through analysis. These two indicators can be used to better analyze the model, so we calculated the output value of the model under the action of these two indicators, as shown in Figure 8. It can be seen from Figure 8 that the two different evaluation indexes have different trends. It can be seen from data changes that the data increase slowly with the increase in iteration number, and the corresponding increase rate decreases gradually, indicating that the slope of data decreases gradually. When the number of iterations increased further, the corresponding test data fluctuated and showed a trend of gradual decline. The mean square error increases gradually with the increase in iteration steps, then tends to be stable, and then shows a trend of gradual decline. With the increase in the number of iterations, the corresponding direction variable first presents a gradually decreasing trend and then a gradually increasing volatility change. Through the analysis, it can be seen that the two indicators can better describe the overall trend of data change. And the variation range of the test data is between the two, so the indicators of the two variables can be comprehensively considered, so as to accurately describe the test data.

## 3. Application of Public Health Art Works Based on Artificial Intelligence Technology

### 3.1. Creation Concept of Art Works

Artistic creation plays an important role in the field of public health, but with the development of society, there are some problems in the field of artistic creation. In order to further analyze and solve these problems, the different concepts of art creation in the field of public health are extracted to obtain different representative indicators: artistic theme, artistic form, artistic content, artistic style, and artistic connotation. The corresponding index change curve is shown in Figure 9. It can be seen from the changes in the figure that artistic indicators can well reflect the specific changes in artistic creation. Through quantitative analysis, it can be seen that the concept value of art theme is about 40, and that of art form is about 20. The concept value of art content is about 10, the concept value of art style is about 30, and the concept value of art connotation is the highest, about 50.

### 3.2. The Application of Artistic Creation Concept in Venice Annual Exhibition

The Venice Biennale has a history of 100 years. The international Visual Art Biennale and the Architecture Biennale are held separately and biennially. They rank alongside Documenta Kassel in Germany and Art Basel in Switzerland as the highest international exhibition of contemporary art. The Venice Architecture Biennale was first held in 1895. In the course of more than 120 years, it has become the most influential event in the world architecture art and academia.

Based on the creation concept of public health visual art works under the effect of artificial intelligence, the algorithm and network model corresponding to the creation of public health visual art works are obtained by considering the artificial intelligence technology and the basic model of the neural network [32, 33]. In order to further study the computational process of visual art works, the flow chart of artistic creation concept based on artificial intelligence technology is analyzed and drawn. It can be seen from Figure 10 that, firstly, the data should be initialized to obtain the corresponding data preprocessing structure, and then, the training set of public health should be verified and analyzed. Secondly, the bidirectional neural network model is constructed, and then, the training and judgment of the network model are used to verify whether the data meet the requirements. If it meets the requirements, it will be imported into the public health visual art test set for visual accuracy monitoring and detection. If it does not meet the requirements, the model parameters should be adjusted and imported into the model training module for further analysis until the requirements are met.

The public health visual art creation concept based on artificial intelligence has a good application in the Venice Biennale [34, 35]. In order to further study and analyze the specific changes of artistic creation concept, the application model of visual art creation is obtained based on artificial intelligence technology, and the corresponding model calculation curve under the effect of artificial intelligence is obtained through calculation, as shown in Figure 11. Through the calculation results, it can be seen that five different artistic creation concepts have different trends: The curve corresponding to the art theme shows a gradual increasing trend with the increase in time, but its increasing range is relatively small. When the corresponding time is 13, the curve appears a certain jump, and then gradually increases. The increase in the corresponding change curve of the art form shows an approximate linear trend of change. In a higher range, the fluctuation range is relatively large. However, with the gradual increase in art content, it shows a trend of gradual decline. When the corresponding time reaches 8, the curve reaches the lowest. With the further increase in time, the corresponding data show a trend of gradual increase, but the range of increase is relatively small. The curves corresponding to artistic styles show a gradually increasing range of variation with the increase in time, and the increasing variables are basically the same, indicating that the linear characteristics of curves are relatively obvious. And the curve corresponding to artistic connotation index shows a trend of gradual decline with the increase in time, with a relatively small range of decline. When the corresponding time reaches 14, the curve drops rapidly and gradually approaches the minimum value.

## 4. Discussion

Based on artificial intelligence technology, the creation model of public health visual art works can be obtained using a neural network basic model and an error backpropagation algorithm. The model can calculate and analyze the application of artistic ideas to the Venice Biennale. In order to further improve and verify the accuracy of the model, the model was used to calculate the creation concept of public health visual art works, so as to obtain the corresponding experimental data and model calculation curve, as shown in Figure 12. As can be seen from the changes of the experimental data in the figure, the data first present a downward trend with the gradual increase in independent variables. When it reaches the local lowest point, the data gradually increase with the increase in independent variables and then gradually decrease. The overall trend is a fluctuation, and the nonlinear characteristics of the data are obvious. The corresponding model calculation curve can not only reflect the trend of data transformation, but also better explain the specific key data. Therefore, the corresponding curve of the model can well reflect the changes of experimental data, which indicates that the public health model based on artificial intelligence technology can be used to analyze the role of artistic creation in the Venice Biennale.

## 5. Conclusion

1. In the change curve of the excitation function, the influence of the threshold value on the output value shows an increasing trend on the whole, and the overall change range is relatively large. The excitation function fluctuates with the increase in input value, and the linear characteristic is obvious.
2. Different parameters have different influences on the function of the error backpropagation algorithm, in which the curve corresponding to the actual value has the largest variation range and the corresponding straight line segment has the highest slope. It shows that the actual value parameter has the greatest influence on the propagation algorithm, while the model value has the least influence on the propagation algorithm.
3. Two different evaluation indicators have different forms of evaluation of test data, among which mean square error can well describe the change trend of test data. However, the specific data of direction variables are higher than the experimental data, so it is necessary to conduct a comprehensive analysis of the two evaluation indicators.

## Figures and Tables

**Figure 1:** Flow chart of neural network training.

**Figure 2:** Excitation function variation diagram.

**Figure 3:** Hebb's learning rule method curve.

**Figure 4:** *ω* learning method curve.

**Figure 5:** Contour map corresponding to the similarity learning method.

**Figure 6:** Function calculation result.

**Figure 7:** Model weight modification variable graph.

**Figure 8:** Calculation chart of different evaluation indexes.

**Figure 9:** Public health art work evaluation concept map.

**Figure 10:** Flow chart of application of artistic creation concept under artificial intelligence technology.

**Figure 11:** Art works with artificial intelligence technology.

**Figure 12:** Model validation curve.

## Data Availability

The experimental data used to support the findings of this study are available from the corresponding author upon request.

## References

[1] Park H. S. (2018). Methodologic guide for evaluating clinical performance and effect of artificial intelligence technology for medical diagnosis and prediction. *Radiology*.

[2] Sun X. (2021). 5G joint artificial intelligence technology in the innovation and reform of university English education. *Wireless Communications and Mobile Computing*.

[3] Yang C. H. (2022). How artificial intelligence technology affects productivity and employment: firm-level evidence from taiwan. *Research Policy*.

[4] Zeba G., Dabic M., Čičak M., Daim T., Yalcin H. (2021). Technology mining: artificial intelligence in manufacturing. *Technological Forecasting and Social Change*.

[5] Zhang F. (2022). Design and implementation of industrial design and transformation system based on artificial intelligence technology. *Mathematical Problems in Engineering*.

[6] Zhang X., Chen L. (2021). College English smart classroom teaching model based on artificial intelligence technology in mobile information systems. *Mobile Information Systems*.

[7] Allareddy V., Min K. L., Vaid N. R. (2021). Use of neural network model to examine post-operative infections following orthognathic surgeries in the United States. *Seminars in Orthodontics*.

[8] Basir M. S., Chowdhury M., Islam M. N. (2021). Artificial neural network model in predicting yield of mechanically transplanted rice from transplanting parameters in Bangladesh. *Journal of Agriculture and Food Research*.

[9] Ding W., Guo X., Wang G. (2021). Radar-based human activity recognition using hybrid neural network model with multi-domain fusion. *IEEE Transactions on Aerospace and Electronic Systems*.

[10] Ghiasi B., Sheikhian H., Zeynolabedin A. (2020). Granular computing-neural network model for prediction of longitudinal dispersion coefficients in rivers. *Water Science and Technology*.

[11] Hmj A., Mte A., Ac A. (2021). An artificial neural network model for multi-pass tool pin varying FSW of AA5086-H34 plates reinforced with Al 2 O 3 nanoparticles and optimization for tool design insight. *CIRP Journal of Manufacturing Science and Technology*.

[12] Joshi V. M., Ghongade R. B., Joshi A. M. (2022). Deep BiLSTM neural network model for emotion detection using cross-dataset approach. *Biomedical Signal Processing and Control*.

[13] Liu Y., Wang X., Tang Z. (2021). Probabilistic ensemble neural network model for long-term dynamic behavior prediction of free-floating space manipulators. *Aerospace Science and Technology*.

[14] Ren L. (2021). Three-dimensional convolutional neural network model for early detection of pine wilt disease using UAV-based hyperspectral images[J]. *Remote Sensing*.

[15] Ma Tovar R., Pérez M. R., Martínez P. . E. R. (2022). Itineraries for charging and discharging a BESS using energy predictions based on a CNN-LSTM neural network model in BCS, Mexico. *Renewable Energy*.

[16] Vu H. L., Ng K., Richter A. (2021). The use of a Recurrent Neural Network model with separated time-series and lagged daily inputs for waste disposal rates modeling during COVID-19. *Sustainable Cities and Society*.

[17] Wang C., Ju Y., Zou Q. (2021). DeepAc4C: a convolutional neural network model with hybrid features composed of physicochemical patterns and distributed representation information for identification of N4-acetylcytidine in mRNA. *Bioinformatics*.

[18] Wlab C., Xin Y. A., Tg A. (2022). Predicting the shelf life of Trachinotus ovatus during frozen storage using a back propagation (BP) neural network model. *Aquaculture and Fisheries*.

[19] Xu S., Feng N., Liu K., Liang Y., Liu X. (2021). A weighted fuzzy process neural network model and its application in mixed-process signal classification. *Expert Systems with Applications*.

[20] Dbh A., Abouda S. E., Medhaffar H. (2021). An improved method for stochastic nonlinear system’s identification using fuzzy-type output-error autoregressive hammerstein–wiener model based on gradient algorithm, multi-innovation, and data filtering techniques. *Complexity*.

[21] Aneja S., Sharma A., Gupta R., Yoo D. Y. (2021). Bayesian regularized artificial neural network model to predict strength characteristics of fly-ash and bottom-ash based geopolymer concrete. *Materials*.

[22] Cui Y., Liu H., Wang Q. (2022). Investigation on the ignition delay prediction model of multi-component surrogates based on back propagation (BP) neural network. *Combustion and Flame*.

[23] Dong W. K., Min S. K., Lee J. (2020). Adaptive learning-rate backpropagation neural network algorithm based on the minimization of mean-square deviation for impulsive noises. *IEEE Access*.

[24] Gautam A., Singh V. (2020). CLR-based deep convolutional spiking neural network with validation based stopping for time series classification. *Applied Intelligence*.

[25] Jin X., Liu Q., Long H. (2020). Impact of cost-benefit analysis on financial benefit evaluation of investment projects under back propagation neural network. *Journal of Computational and Applied Mathematics*.

[26] Liu X., Ke Z., Chen Y. (2022). The feasibility of designing a back propagation neural network to predict the levitation force of high-temperature superconducting magnetic levitation. *Superconductor Science and Technology*.

[27] Liu Y. B., Ying-Li W., Zhang W. (2020). Design of small solar power generation system based on GA-BP prediction algorithm. *Sensor World*.

[28] Sogabe T. (2021). Quantum circuit learning with error backpropagation algorithm and experimental implementation. *Quantum Reports*.

[29] Tian J., Xie J., He Z. (2021). A device employing a neural network for blood pressure estimation from the oscillatory pressure pulse wave and PPG signal. *Sensor Review*.

[30] Wang J., Yang B., Li D. (2021). Photovoltaic cell parameter estimation based on improved equilibrium optimizer algorithm. *Energy Conversion and Management*.

[31] Zhang M., Wang J., Zhang Z. (2020). Spike-timing-dependent back propagation in deep spiking neural networks. *arXiv*.

[32] Fujii H., Managi S. (2018). Trends and priority shifts in artificial intelligence technology invention: a global patent analysis. *Economic Analysis and Policy*.

[33] Khanagar S. B., Al-Ehaideb A., Vishwanathaiah S. (2020). Scope and performance of artificial intelligence technology in orthodontic diagnosis, treatment planning, and clinical decision-making - a systematic review. *Journal of dental sciences*.

[34] Leonov P., Kozhina A., Leonova E., Epifanov M., Sviridenko A. (2020). Visual analysis in identifying a typical indicators of financial statements as an element of artificial intelligence technology in audit. *Procedia Computer Science*.

[35] Li J., Yang Y., Ren Z. (2021). Design of higher education system based on artificial intelligence technology. *Discrete Dynamics in Nature and Society*.

